# Low-Dose X-Ray Increases Paracellular Permeability of Human Renal Glomerular Endothelial Cells

This article has been retracted.

**DOI:** 10.1155/2022/5382420

**Published:** 2022-10-11

**Authors:** Jilei Wang, Chongtao Sun, Dongxia Zheng, Kun Sun

**Affiliations:** ^1^Department of Nephrotic Diagnosis and Treatment Center, The Second Affiliated Hospital of Shandong University of Traditional Chinese Medicine, No. 1 Jingba Road, Shizhong District, Jinan, Shandong 250001, China; ^2^Department of Nephrology, Zibo First Hospital, No. 4 Emeishandong Road, Boshan District, Zibo, Shandong 255200, China; ^3^Department of Nephrology, Dongying People's Hospital, No. 317 Nanyi Road, Dongying, Shandong 257091, China; ^4^Department of Nephropathy, Shandong Zibo Central Hospital, No. 54 Gongqingtuanxi Road, Zhangdian District, Zibo, Shandong 255036, China

## Abstract

**Objective:**

Glomerular endothelium functions as a filtration barrier of metabolites in the kidney. Although X-ray irradiation modulated the permeability of the vascular endothelium, the response of human renal glomerular endothelial cells (HRGECs) to low-dose X-ray irradiation has not been investigated. We evaluated the impacts of low-dose X-ray irradiation on HRGECs and revealed the underlying mechanism.

**Methods:**

HRGECs were exposed to X-ray with doses of 0, 0.1, 0.5, 1.0, and 2.0 Gy. The proliferation, viability, and apoptosis of HRGECs were examined by MTT assay, trypan blue staining assay, and TUNEL staining, respectively. The paracellular permeability was assessed by paracellular permeability assay. The expression of VE-cadherin was investigated via immunofluorescence assay. Western blot and qRT-PCR detected the expression levels of VE-cadherin and CLDN5. Besides, the expression levels of pVE-cadherin (pY658), TGF-*β*, TGF-*β*RI, Src, p-Src, Smad2, p-Smad2, Smad3, p-Smad3, SNAIL, SLUG, and apoptosis-related proteins were tested by Western blot.

**Results:**

The proliferation, viability, and apoptosis of HRGECs were not affected by low-dose (<2.0 Gy) X-ray irradiation. X-ray irradiation dose-dependently reduced the level of VE-cadherin, and VE-cadherin and CLDN5 levels were reduced with X-ray irradiation. The levels of pY658, p-Src, p-Smad2, and p-Smad3 were upregulated with the increase in X-ray dose. Besides, the paracellular permeability of HRGECs was increased by even low-dose (<2.0 Gy) X-ray irradiation. Therefore, low-dose X-ray irradiation reduced the cumulative content of VE-cadherin and increased the level of pY658 via activation of the TGF-*β* signaling pathway.

**Conclusion:**

Even though low-dose X-ray exposure had no impact on proliferation, viability, and apoptosis of HRGECs, it increased the paracellular permeability by deterioration and downregulation of VE-cadherin through stimulating the TGF-*β* signaling pathway. This study built the framework for kidney response to low-dose irradiation exposure.

## 1. Introduction

The glomerulus, located at the end of each nephron in the kidney, is a ball of capillaries and is involved in the process of blood filtration for urine formation [1]. Generally, filtration function is achieved by 3 components: glomerular endothelial cells (GECs), glomerular basement membrane, and epithelial cells of Bowman's capsule (surround the glomerulus) [2]. Herein, the impaired GECs are commonly associated with acute and chronic kidney diseases, along with systemic lesions.

VE-cadherin is a transmembrane protein mediating cell adhesion and vascular permeability [3, 4]. Two VE-cadherins can form a homomeric dimer between cells. Besides, VE-cadherin can regulate the rearrangement of the cytoskeleton via interaction with intracellular catenin [5, 6]. The inflammation of the glomerulus caused by high pressure, viral infection, antibiotic administration, or ionizing radiation changes the paracellular permeability of GECs through VE-cadherin cleavage [7–9]. Studies have shown that claudin 5 (CLDN5) is a major integral membrane protein involved in proper tight junctions [9] and its expression level has a negative correlation with cells' permeability which is involved in the maintenance of microvascular integrity of endothelial cells [10, 11].

X-ray, or X-irradiation, is a type of high-energy electromagnetic radiation. Currently, X-ray is widely used for medical imaging and radiotherapy. The risk of X-ray is due to the low dose (from 0.1 mGy to 400 mGy) applied [12, 13]. However, long-time and high-dose X-ray exposures have adverse impacts on human health by affecting cell biological processes [12]. In contrast, low-dose X-ray exposures were reported to have limited or rare detrimental effects on cell viability of human dermal lymphatic endothelial cells (HDLECs), while it promotes the rearrangement of cytoskeleton and alters the intercellular junctions mediated by VE-cadherin to enhance the paracellular permeability of HDLECs [13, 14].

Li and Jimenez found that VE-cadherin of TGF-*β* treatment endothelial cells downregulated significantly, indicating that the TGF-*β* signaling pathway negatively regulated VE-cadherin expression [15]. Besides, the activation of the TGF-*β* signaling pathway induced high permeability of human renal GECs (HRGECs) via upregulation of the downstream Smad proteins (such as Smad2 and Smad3) [16, 17]. It has been proved that TGF-*β* is activated through binding to T*β*R-II to form a heterodimer. Then, the heterotrimer of T*β*R-II/TGF-*β*/T*β*R-I is formed by recruitment of T*β*R-I to stimulate the phosphorylation of Smad proteins [18, 19]. Nagaharu et al. have demonstrated that phosphorylation of Src is significantly upregulated with the activation of TGF-*β* [20]. Src-controlled cytoskeleton and cell migration and increased Src activity are related to the pathogenesis of renal tumors and certain glomerular diseases [21]. Phosphorylated Src promotes the phosphorylation of VE-cadherin at Tyr658 (pY658). Besides, phosphorylation of VE-cadherin in the cytoplasmic results in the deficiency of VE-cadherin at endothelial junctions [22, 23]. In addition, SNAIL and SLUG are important regulators of cytoskeletal stability, which mainly induce epithelial-mesenchymal transition (EMT) [24, 25].

Hence, we investigated whether low-dose X-ray has an impact on the permeability of HRGECs without affecting cell proliferation and apoptosis. Besides, the underlying mechanism was also explored via the analysis of the expression of VE-cadherin mediated by the TGF-*β* signaling pathway.

## 2. Materials and Methods

### 2.1. Cell Culture

Primary HRGECs were purchased from ScienCell (USA) and incubated in ECM (ScienCell, USA) containing 5% FBS, 1% endothelial cell growth supplement, and 1% p/s in a humidified incubator with 5% CO_2_ at 37°C.

### 2.2. X-Ray Irradiation

HRGECs from passages 2–4 were expanded in the monolayer in the new culture vessels. When reaching 90% confluence, the culture medium was substituted by FBS-free solution 24 h before the subsequent experiment (starvation step). Then, the cells were exposed to 0, 0.1, 0.5, 1, and 2 doses of X-ray using a Varian 21EX Linear Accelerator operating at a photon energy of 6 MV. The X-ray dose rate was 2.0 Gy/min.

### 2.3. MTT Assay

The irradiated HRGECs (resuspended in standard ECM) were seeded in a 96-well plate at a density of 5 × 10^3^–10^4^ cells per well and incubated for 7 days. Then, the cells were replenished by FBS-free ECM containing 0.5 mg/mL MTT solution. After incubation for 4 h, the media were removed and 150 *μ*L of DMSO was added. The crystal was dissolved and the absorbance was measured at OD_570_.

### 2.4. Trypan Blue Staining

The HRGECs (resuspended in FBS-free ECM) were mixed with 0.4% trypan blue at a ratio of 1 : 1 (*v*/*v*). The mixture was incubated for 3 min, and the cells were counted in a hemocytometer using the inverted microscope CKX53 (Olympus, Japan).

### 2.5. TUNEL Assay

The One-Step TUNEL Apoptosis Assay Kit (Beyotime, China) was used. 7 days after X-ray irradiation, the cells were washed with PBS (pH 7.4) and then fixed with 4% paraformaldehyde for 0.5 h. Then, the cells were incubated with PBS containing 0.1% Triton X-100 on ice. After being washed, the cells were incubated with TUNEL detection solution for 1 h. DAPI was used for nuclear staining, and the dyed cells were photographed using CKX53 microscopy (Olympus, Japan).

### 2.6. qRT-PCR

The RNAs were extracted using TRIzol (Invitrogen, USA). The cDNAs were reversed from total RNAs by the RevertAid First Strand cDNA Synthesis Kit (Thermo Fisher, USA). qRT-PCR was performed using a LightCycler® 480 II real-time PCR instrument (Roche, Switzerland) and SYBR Green PCR mix (Beyotime, Chian). GAPDH served as the internal control. Primers were used as follows: VE-cadherin forward primer: 5′-CCAAAGTGTGTGAGAACGCT-3′; reverse primer: 5′-CGTTTCGTGGT GTTATGTCC-3′; CLDN5 forward primer: 5′-GACCTTCTCCTGCCACTAT-3′; reverse primer: 5′-CGCTCTGCCTATGGAAAC-3′; GAPDH forward primer: 5′-TGATGACATCAAGAAGGTGGTGAAG-3′; reverse primer: 5′-TCCTTGGAGGCCATGTGGGCCAT-3′.

### 2.7. Western Blot

The cells were lysed by RIPA (Thermo Fisher, USA) and proteins were quantified by the BCA kit (Thermo Fisher, USA). The lysates were separated by 12% SDS-PAGE and transferred onto PVDF membranes. After being blocked and washed, the primary antibodies against human VE-cadherin, phospho-VE-cadherin, CLDN5, Bax, Bcl-2, cleaved caspase 3, TGF-*β*RI, Smad2, p-Smad2, Smad3, p-Smad3, Src, phospho-SRC, SNAIL, SLUG, and GAPDH (Abcam, USA) were applied. Next, the membranes were incubated with the corresponding HRP-labeled secondary antibodies for 1 h. The blots were detected with the SuperSignal Chemiluminescent Kit (Thermo Fisher, USA). The intensities were measured by ImageJ.

### 2.8. Paracellular Permeability

The *In Vitro* Vascular Permeability Assay Kit (24 wells, cat. #ECM644, Millipore) was used to evaluate the paracellular permeability of HRGECs. Briefly, 200 *μ*L of HRGEC suspension was seeded into the inserts (1 *μ*m pores within a polyethylene terephthalate membrane) at a density of 1 × 10^5^ cells per insert. 500 *μ*L of standard ECM was added to the receiver plate well. The cells were then incubated until a monolayer was formed. Then, the cells were subjected to starvation and irradiation (see above). Seven days after irradiation, the media in the inserts were replaced with FBS-free ECM comprising 1 mg/mL FITC-dextran with 50 kDa and the cells were incubated for 0.5 h. During this time, FITC-dextran would translocate from the inserts to the receiver plate wells. Then, media from receiver plate wells were collected and transferred to black 96-well plates. The fluorescence was measured using a plate reader.

### 2.9. Immunofluorescence Assay

The cells were rinsed with PBS and fixed with 4% paraformaldehyde. After being washed and sealed, the cells were treated with the anti-VE-cadherin antibody (Abcam, USA) overnight at 4°C. Then, the FITC-labeled secondary antibody (Abcam, USA) was applied. DAPI was used for nuclear staining, and the cells were photographed using the CKX53 microscope (Olympus, Japan).

### 2.10. Statistical Analysis

Statistical significance was evaluated using Student's *t*-test or one-way analysis of variance (ANOVA) by SPSS 18.0. *P* < 0.05 was considered a significant difference. All experiments were repeated three times unless otherwise stated.

## 3. Results

### 3.1. Low-Dose X-Ray Irradiation Does Not Affect the Proliferation and Viability of HRGECs

HRGECs were cultured until confluence to allow for the formation of proper cell junctions. The cells were then irradiated with 0, 0.1 0.5, 1.0, and 2.0 Gy doses of X-ray. Seven days after irradiation, no significant difference in cell proliferation was observed under low-dose X-ray treatments by MTT assay (Figure 1(a)). Besides, the results of trypan blue staining showed that low-dose (<2.0 Gy) X-ray irradiation did not affect the viability of HRGECs (Figure 1(b)). These results above demonstrated that HRGECs could tolerate low-dose X-ray irradiation.

### 3.2. Low-Dose X-Ray Irradiation Does Not Affect the Apoptosis of HRGECs

Long-time and high-dose X-ray exposures were known to induce DNA double-strand breaks and activate cell apoptosis. In this study, the HRGECs were treated with various doses of X-rays. The result of TUNEL showed that low-dose (<2.0 Gy) X-ray irradiation did not change the percentage of apoptotic cells (Figure 2(a)). Furthermore, the results of Western blot showed that there was no significant difference in the expression levels of apoptosis-related proteins in the groups with low-dose (<2.0 Gy) X-ray treatments and the control group (Figures 2(b)–2(d)). Therefore, the apoptosis of HRGECs was not affected by low-dose X-ray irradiation.

### 3.3. X-Ray Irradiation Increases the Paracellular Permeability of HRGECs

FITC-dextran of 50 kDa was used to test the paracellular permeability of HRGECs in the paracellular permeability assay. Low-dose X-ray exposure significantly increased the paracellular permeability of FITC-dextran X-ray dose dependently (Figure 3(a)). The cell-cell junctions were critical for keeping paracellular permeability, so we investigated whether X-ray irradiation disrupted the integrity of cell junctions. VE-cadherin, a major component for cell junctions, was detected by immunofluorescence staining (Figure 3(f)). Furthermore, the expression levels of VE-cadherin (Figures 3(d) and 3(e)) and CLDN5 (Figures 3(b) and 3(c)) protein and mRNA levels were also decreased by X-ray dose dependently. The results showed that VE-cadherin and CLDN5 were decreased in an X-ray dose-dependent manner. All results above suggested that low-dose X-ray exposure could increase the paracellular permeability of HRGECs via inhibition of the expression levels of VE-cadherin and CLDN5.

### 3.4. X-Ray Irradiation Activates the TGF-*β* Signaling Pathway in HRGECs

Previous studies had demonstrated that the VE-cadherin level was regulated by the TGF-*β* signaling pathway [19, 20, 22, 23, 26], which encouraged us to investigate whether X-ray irradiation could stimulate the TGF-*β* signaling pathway in HRGECs. After X-ray irradiation, the phosphorylation levels of Smad2, Smad3, and Src were raised, whereas the protein levels of Smad2 and Smad3 were not affected by the doses of X-ray (Figures 4(a)–4(c)), which indicated that the TGF-*β* downstream signaling pathways of TGF-*β*/Smad2/Smad3 and TGF-*β*/Src were activated by the X-ray irradiation. Moreover, the expression levels of TGF-*β*RI, SNAIL, SLUG, and pY658 involved in the TGF-*β* signaling pathway were upregulated in an X-ray dose-dependent way (Figure 4(d)). Thus, the downregulated expression level of VE-cadherin was related to the increased phosphorylated levels of Src, Smad2, Smad3, and VE-cadherin mediated by the activation of the TGF-*β* signaling pathway. Hence, we concluded that X-ray irradiation inhibited the expression of VE-cadherin via activation of the TGF-*β* signaling pathway in HRGECs.

## 4. Discussion

Long-time and high-dose X-ray exposures cause mutations of DNA and therefore lead to cancer. However, the limited adverse health effects of exposure to transient and low-dose X-rays are less known. Currently, X-ray irradiation is widely used in radiography, fluoroscopy, and computed tomography. In this study, we found that the proliferation, viability, and apoptosis of HRGECs were not disturbed by low-dose X-ray irradiation. Nevertheless, the paracellular permeability of HRGECs was increased by X-ray irradiation. Therefore, low-dose X-ray exposures might have an impact on the permeability and filtration function of the kidney.

Low-dose X-ray affects cellular functions. Wu et al. have studied the roles of low-dose ionizing radiation (LDIR) on stem cells [27]. LDIR disrupts the metabolism of hippocampal glial cells, causing inflammatory responses and the release of inflammatory factors [28]. LDIR activates MAPK/ERK and PI3K/AKT signaling pathways in human embryonic lung fibroblasts [29]. The permeability of endothelium can be influenced by various external factors such as interleukin-1*β* (IL-1*β*), MAPK, and cadmium (Cd) through a variety of signaling pathways [30–32]. IL-1*β* is overexpressed and secreted into the circulatory system through the TGF-*β*-mediated NF-*κ*B pathway and interacts with the vascular endothelium to increase vascular permeability [33]. It has been proved that a low dose of Cd induces the dispersion of VE-cadherin and p38 MAPK mediates Cd-induced disruption of endothelial cell barrier function and promotes increased vascular permeability [34]. TGF-*β* has been also found to increase endothelial permeability through activating Smad2-dependent p38 and downstream factor RhoA [33]. In addition, the activation of Src-dependent pathways promotes VE-cadherin phosphorylation, destroys VE-cadherin/*β*-catenin binding, and transfers VE-cadherin to the cytoplasm, leading to increased permeability [35, 36]. The Western blot results in Figure 4 suggested the expression level of pY658 was upregulated by the activated Src through the TGF-*β*/Smads signaling pathway. Moreover, the phosphorylation of Y658 damaged the stability of tight connections by suppressing the combination of p120 and VE-cadherin [37].

The downregulation of VE-cadherin expression caused by TGF-*β* which was activated by low-dose X-ray indicated the negative correlation between TGF-*β* and VE-cadherin [38]. Furthermore, TGF-*β* was recently reported to increase the permeability of vascular endothelial monolayers via tyrosine phosphorylation of VE-cadherin and upregulation of matrix metalloproteinase-9 (MMP-9) [21, 38]. Besides, two downstream factors SNAIL and SLUG involved in the TGF-*β* signaling pathway were reported to bind to the promoter of VE-cadherin and subsequently suppress the expression of VE-cadherin [39]. Thus, the content of VE-cadherin was reduced via downregulation of VE-cadherin and increase of the tyrosine phosphorylation level of VE-cadherin, which leads to the broke cytoskeleton stability and increased paracellular permeability. Our study further revealed that low-dose X-ray exposures increased the paracellular permeability of HRGECs caused by deterioration and downregulation of VE-cadherin expression. Therefore, the proposed underlying mechanism is that low-dose X-ray irradiation stimulates the TGF-*β* signaling pathway without affecting cell growth. This stimulation process was followed by the inhibition of VE-cadherin, which leads to the break of cell-cell junctions and increased the paracellular permeability of cells.

In summary, this study exhibited that low-dose X-ray exposures increase the paracellular permeability of HRGECs through inhibition of the expression level of VE-cadherin by activating the TGF-*β* signaling pathway. This study implies that low-dose X-ray exposures might affect the function of the glomerular filtration barrier, which is related to a variety of kidney diseases. The mechanism by which TGF-*β* responds to irradiation and how TGF-*β* modulates the cleavage or expression of VE-cadherin need further exploration.

## Figures and Tables

**Figure 1:** The proliferation and viability of HRGECs under different doses of X-ray. The proliferation percentage by MTT assay (a) and viability percentage by trypan blue staining (b). The percentage of proliferation and viability showed no significant difference in low-dose X-rays (<2.0 Gy).

**Figure 2:** Low-dose X-ray irradiation does not affect the apoptosis of HRGECs. The apoptosis of HRGECs was detected by TUNEL apoptosis assay (a). Besides, Western blot bands of Bcl-2 (b), Bax (c), and cl-casp-3 (d) were statistically analyzed and GAPDH was used as an internal control. It was obvious that the apoptosis was consistent under low-dose X-ray (<2.0 Gy).

**Figure 3:** X-ray irradiation increases the paracellular permeability of HRGECs through the disruption of cell junctions. HRGECs was cultured for seven days under 0, 0.1, 0.5, 1.0, and 2.0 Gy X-ray irradiation. 50 kDa FITC-dextran was used to determine the permeability of HRDECs (a). The transfer amount of 50 kDa FITC-dextran across the HRGECs monolayer without X-ray irradiation was set to 1. Western blot bands of CLDN5 (b) and VE-cadherin (d) were tested and analyzed. GAPDH was used as an internal control. The mRNA results of CLDN5 (c) and VE-cadherin (e) were detected by qRT-PCR. Immunofluorescence images of cell junctions (f) were shown by staining VE-cadherin with fluorescent antibodies (green), and DAPI was used for nuclear staining (blue). ^∗^*P* < 0.05; ^∗∗^*P* < 0.01.

**Figure 4:** Western blot analysis of proteins involved in the TGF-*β* signaling pathway. GAPDH was used as an internal control. The Western blot results and the corresponding statistical histograms of p-Samd2/Smad2 (a), p-Smad3/Smad3 (b), and p-Src/Src (c) were shown. Besides, the expression levels of TGF-*β*RI, SNAIL, SLUG, and pY658 were detected by Western blot and analyzed by histograms as well. ^∗^*P* < 0.05 and ^∗∗^*P* < 0.01; ^#^*P* < 0.05 and ^##^*P* < 0.01; ^$^*P* < 0.05 and ^$$^*P* < 0.01; ^&^*P* < 0.05 and ^&&^*P* < 0.01.

## Data Availability

The datasets used and/or analyzed during the current study are available from the corresponding author upon reasonable request.

## Additional Points

*Highlights.* (1) The proliferation, viability, and apoptosis of HRGECs are not affected by low-dose X-ray irradiation. (2) Low-dose X-ray irradiation increases the paracellular permeability of HRGECs. (3) Low-dose X-ray irradiation inhibits the expression of VE-cadherin via activation of the TGF-*β* signaling pathway.
